This article has been retracted.

# A Rare Surgical Case of Isolated Double-Chambered Right Ventricle Without Cardiac Malformations in an Older Female Patient

**DOI:** 10.7759/cureus.74051

**Published:** 2024-11-19

**Authors:** Yuki Hayashi, Shunji Osaka, Satoshi Unosawa, Masashi Tanaka

**Affiliations:** 1 Cardiovascular Surgery, Nihon University School of Medicine, Tokyo, JPN; 2 Cardiovascular Surgery, Akabane Central General Hospital, Tokyo, JPN; 3 Cardiovascular Surgery, Unosawa Clinic, Chiba, JPN

**Keywords:** adult surgical case of dcrv, dcrv without congenital heart disease, dcrv without vsd, double-chambered right ventricle (dcrv), elderly surgical case of dcrv

## Abstract

Double-chambered right ventricle (DCRV) is a congenital heart disease. Most cases of DCRV are complicated by another congenital cardiac anomaly. Mostly, a ventricular septal defect (VSD) is the usual comorbidity. The flow turbulence by VSD has been suggested to be associated with DCRV, which occurs in many patients during childhood, but very rarely in later years of life. Although there are some cases of DCRV in older adults, there is almost no literature on patients over 70 years of age. We report the surgical case of a 72-year-old female patient with isolated DCRV who visited the hospital due to fatigue. Transthoracic echocardiography (TTE) revealed severe right heart overload, severe tricuspid valve regurgitation, and right ventriculography, leading to a diagnosis of DCRV. We resected anomalous muscle bundles caused by right ventricular outflow tract (RVOT) stenosis via the transventricular approach, closed RVOT using a bovine pericardium patch, and performed tricuspid annuloplasty. Intraoperative findings showed no VSD. After surgery, right ventricular pressure decreased significantly, the patient was discharged on postoperative day 20. DCRV is one of the pathological conditions of which prognosis can be improved with appropriate surgical intervention even in advanced age.

## Introduction

The major lesions that cause right ventricular outflow tract (RVOT) stenosis affect the pulmonary valve, infundibulum, and upper part of the pulmonary valve. However, double-chambered right ventricle (DCRV) is a special case. Although DCRV is a relatively common disease in children, as reported by Keith, it is rare in adults [1]. DCRV is thought to be triggered by abnormal muscle bundles in the moderator band and is also associated with an abnormally short distance from a pulmonary artery, and the stenosis progresses over time [2]. On auscultation, a systolic murmur is heard, and as the stenosis progresses, the right ventricle becomes enlarged and cyanosis occurs in cases with VSD [2]. The diagnosis of DCRV can be usefully assessed by the pressure gradient in the right ventricular outflow tract on transthoracic echocardiography (TTE) and morphologically on magnetic resonance imaging (MRI) [3]. Most cases of DCRV are complicated by another cardiac anomaly such as ventricular septal defect (VSD) or patients with repaired tetralogy of Fallot [4]. However, the present case is extremely rare as the patient was 70 years old and had no associated cardiac malformations.

## Case presentation

A 72-year-old female patient with a chief complaint of general malaise for six months visited another hospital and was found to have a heart murmur. On physical examination, a systolic murmur was observed at the left margin of the second intercostal sternum, without total systolic murmur. Chest X-ray radiography revealed an enlarged cardiac-thoracic ratio of 54% without evidence of pulmonary congestion (Figure 1). Blood test results showed N-terminal pro-B-type natriuretic peptide (NT-proBNP) of 1424 pg/mL (Table 1). TTE showed a maximum RVOT flow velocity of 6.0 m/s, a maximum pressure gradient of 147 mmHg (Figure 2), and moderate-to-severe tricuspid valve regurgitation. Cardiac MRI and right ventriculography were performed, and a diagnosis of DCRV was made (Figure 3).

**Figure 1:** Preoperative chest X-ray

**Table 1:** Preoperative NT-proBNP value NT-proBNP: N-terminal pro-B-type natriuretic peptide

Parameter	Normal range	Patient's result
NT-proBNP (pg/mL)	<125	1424

**Figure 2:** Transthoracic echocardiography showing a maximum RVOT flow velocity of 6.0 m/s and maximum pressure gradient of 147 mmHg RVOT: right ventricular outflow tract

**Figure 3:** Cardiac magnetic resonance imaging (A) and right ventriculography (B) showing right ventricular outflow tract obstruction without stenosis of the pulmonary valve (white arrow)

No other cardiac malformations including VSD were observed. The patient was scheduled to undergo RVOT plication and tricuspid valve annuloplasty, wherein the approach to the RVOT was considered from the right atrium but was performed from the anterior right ventricle due to poor visual field. After total cardiopulmonary bypass, an incision just below the RVOT in the anterior right ventricle revealed marked thickening of the ventricular septum just below the pulmonary valve with abnormal muscle bundles (Figure 4).

**Figure 4:** View from the surgical assist's side (right side is cephalad): an incision on the right ventricular myocardium immediately above the right ventricular outflow tract from the anterior surface of the right ventricle reveals an abnormal muscle bundle (A, white arrow); resection of the muscle bundles is performed, and the outflow tract is enlarged and patched (B)

The RVOT was resected as much as possible, and an enlarged RVOT was reconstructed using a bovine pericardial patch. Subsequently, tricuspid valve annulus formation was performed with a flexible ring. The operative time was three hours and 11 minutes. The extracorporeal circulation time was one hour and 38 minutes. Regarding the postoperative TTE, the RVOT maximum pressure gradient was 22 mmHg, and tricuspid regurgitation had subsided completely. Postoperative cardiac MRI also showed that the morphological stenosis of the RVOT had resolved (Figure 5).

**Figure 5:** Postoperative cardiac magnetic resonance imaging showing an enlarged right ventricular outflow tract (white arrow)

The postoperative course was good; the patient was discharged on postoperative day 18. Currently, she is eight years postoperative and has not developed right heart failure.

## Discussion

DCRV is defined as a division of the right ventricle into a high-pressure part on the tricuspid valve side and a low-pressure part on the pulmonary artery valve side by an abnormal muscle bundle that develops below the funnel area [5]. It is a relatively infrequent disorder, accounting for approximately 1% of congenital heart disease [6]. DCRV is often associated with other cardiac malformations, especially VSD, which occurs in approximately 80% of cases [7] and rarely occurs alone [8]. Abnormal muscle bundles that are considered the main cause of this disease develop with age, and subjective symptoms appear with an increase in pressure differential. Therefore, early surgery is essential. Most cases occur in childhood or young adulthood; the occurrence of this disease in older patients over 70 years of age is extremely rare.

In this case, there was no concomitant cardiac malformation, and the hemodynamic status was the same as pulmonary arteriovenous stenosis, which may have been the main reason why the patient remained asymptomatic until over 70 years of age. Abnormal muscle bundles in the DCRV are considered one of the repair mechanisms for VSDs [9,10]; they develop with age, gradually increasing the pressure gradient. Although assuming that the abnormal muscle bundles develop after the spontaneous closure of the VSD is natural, whether they appear at the advanced age of 70 years is unclear. There are two surgical approaches: the right ventriculotomy and the right atrial approach. We considered the right atrial approach for additional treatment of tricuspid regurgitation. However, we had to incise the anterior surface of the right ventricle due to poor visual field. The right ventricular approach is considered to have complications of right ventricular dysfunction and ventricular arrhythmias, but in this case, the right ventricular approach was unavoidably chosen because of the difficulty of approaching from the right atrium. Fortunately, the patient had a good postoperative course without dysfunction of the right ventricle and arrhythmia. A similar direction using patch enlargement of the anterior right ventricular surface may be chosen in the tetralogy of Fallot. Other options include radial balloon dilation, but in cases such as the present case, where the pressure gradient is severe, surgery is the better option. Other complications include restenosis and pulmonary atresia, both of which are common in patients with complicated malformations and pulmonary artery stenosis in which the pulmonary valve is involved [4].

## Conclusions

Although DCRV in older adults is extremely rare, the pathogenesis is not very complicated. A good course is achieved if the RVOT is reliably diagnosed and stenosis of the RVOT is released. In cases of DCRV without congenital cardiac malformations, the mechanism of origin of RVOT is not clear, and aggressive intervention in cases with preserved cardiac function and tolerability would improve the patient's prognosis.
